This article has been retracted.

# Abnormal Plasma Levels of Steroids and Their Ratios in Patients With Prurigo Nodularis: A Pilot Study

**DOI:** 10.3389/fphys.2022.835269

**Published:** 2022-06-28

**Authors:** Liuxi Chu, Xin Shu, Yan Wu, Haoran Yang, Qin Lu, Huihua Deng

**Affiliations:** ^1^ School of Biological Sciences and Medical Engineering, Southeast University, Nanjing, China; ^2^ Key Laboratory of Child Development and Learning Science (Southeast University), Ministry of Education, Nanjing, China; ^3^ Institute of Child Development and Education, Southeast University, Nanjing, China; ^4^ Department of Dermatology, The Third Medical Centre of Chinese PLA General Hospital, Beijing, China; ^5^ Department of Prescription Science, School of Basic Medical Sciences, Hebei University of Chinese Medicine, Shijiazhuang, China

**Keywords:** prurigo nodularis, cortisol, cortisone, dehydroepiandrosterone, pruritus severity

## Abstract

**Background:** It has been suggested that cortisol levels are abnormal in chronic urticaria and atopic dermatitis, but other steroids, such as dehydroepiandrosterone (DHEA) and testosterone, are still unknown, and whether these hormones affect the maintenance of skin homeostasis or the pathogenesis of skin diseases is not fully understood. Limited data are available on steroid levels in prurigo nodularis (PN)-related research, and no study has examined the association between pruritus severity and steroid levels in PN patients.

**Aims:** This pilot study aimed to investigate the differences in the levels of five steroids combined with their ratios in plasma between PN patients and controls and to examine the associations between the biomarkers and pruritus severity.

**Methods:** Plasma concentrations of five steroids, including cortisol, cortisone, testosterone, progesterone, and dehydroepiandrosterone (DHEA), in 36 patients with PN were compared with concentrations in thirty-six and matched healthy controls. The concentrations of steroids were quantitated using liquid chromatography-tandem mass spectrometry. The PN symptoms, including pruritus severity, pain, and life quality, were assessed with the use of the visual analog scale, prurigo score index, numerical rating scale, and verbal rating scale and dermatology life quality index scores.

**Results:** In comparison with controls, PN patients had lower levels of plasma cortisol and cortisone, which negatively correlated with PN symptoms. PN patients had higher levels of cortisone and testosterone to cortisol, which positively correlated with pruritus severity. Additionally, there were no significant differences in plasma concentrations of DHEA and testosterone between the two groups. We found no correlation between plasma concentrations of DHEA and testosterone and pruritus severity.

**Conclusion:** This pilot study suggests that there may be abnormalities in peripheral blood levels of cortisol, and cortisone and the ratios of cortisone and testosterone to cortisol in patients with PN, and they are related to pruritus severity. The plasma concentrations of testosterone and DHEA may be not abnormal in PN patients and may not be associated with pruritus severity.

## 1 Introduction

Prurigo nodularis (PN) is a chronic inflammatory skin disease characterized by multiple intensely pruritic, papulonodular lesions occurring in the background of intense pruritus with unknown causes, mechanisms and mediators (Sonkoly et al., 2006; Ständer et al., 2020). Dysfunction of the neuroendocrine-immune system due to stress may play a critical role in the pathogenesis of PN. Psychological stress appears to play a significant role in PN, as studies have found a correlation between stress and the deterioration of symptoms (Schneider et al., 2006; Brenaut et al., 2019). Indeed, most studies have shown that the symptoms of anxiety and depression in patients with PN are more serious than those in healthy controls (Jørgensen et al., 2017; Brenaut et al., 2019). However, in previous studies, the stress-related assessment of PN patients was usually based on a self-report psychological questionnaire (Dazzi et al., 2011; Dalgard et al., 2015; Oh et al., 2015; Schut et al., 2016; Jørgensen et al., 2017; Pölking et al., 2018; Brenaut et al., 2019; Chen et al., 2019). Despite their simplicity and affordability, self-reported psychometric methods lack objectivity, leading to overestimation of stress-induced PN symptoms. Therefore, it is urgently necessary to investigate the physiological responses associated with PN, so that objective biomarkers can be developed to comprehensively assess the stress response of PN.

Cortisol and cortisone are secreted by the hypothalamic pituitary adrenal (HPA) axis in response to stress, which is one of the main stress-sensitive systems and adjusts the body’s adaptation (Papadimitriou and Priftis, 2009; Kim et al., 2013; Kino, 2015). Although there is no empirical study on the physiological response of PN, some inspiration can be obtained from similar chronic skin diseases such as atopic dermatitis (AD). A common pathogenesis of AD and PN was suggested by previous observations of dermal hyperplasia of nerve fibers or increased skin levels of interleukin 31 (IL-31) in both PN and AD (Sugiura et al., 1997; Sonkoly et al., 2006). Cortisol reduces the secretion of IL-4 and IL-5, which are stimulating factors in the early stage of AD, and it has been shown that AD patients have lower stress-induced cortisol production than healthy controls (Buske-Kirschbaum et al., 2010). In addition, the role of cortisol in the pathogenesis of chronic skin diseases is also discussed. For instance, patients with chronic urticaria showed lower concentrations of cortisol and dehydroepiandrosterone sulfate, which is a metabolite of dehydroepiandrosterone (DHEA) (Sonia Louise and Robin, 2006) than healthy controls (Brzoza et al., 2008; Varghese et al., 2016), which was attributed to the fact that the activity of the HPA axis was fatigued under long-term chronic itching stress. However, the importance of cortisol in PN has not yet been determined.

Moreover, limited data are available on employing the concentrations of DHEA, testosterone and progesterone, which are secreted by the hypothalamo-pituitary-gonadal (HPG) axis (Chu et al., 2020; Zavala et al., 2020; Chu et al., 2021), in skin disease-related research, and no study has examined these concentrations of sex steroids in PN patients. To date, no study has investigated the activities of the HPA and HPG axes in PN patients, and a few studies have examined the association between pruritus severity and steroid levels in PN patients. Moreover, dysfunction of the neuroendocrine-immune system was observed in the presence of skin diseases as previously described. Studies have shown that some changes in the metabolism and balance of glucocorticoids and sex hormones may be susceptible factors of immune-mediated diseases (Kasperska-Zajac et al., 2007; Vinnik et al., 2020). It has been shown that glucocorticoids, such as cortisol and cortisone, and sex steroids, such as DHEA and testosterone, have multiple immunomodulatory effects (Bereshchenko et al., 2018). For example, DHEA may affect the balance between type 1 and type 2 helper T cells (Th1/Th2), immunoglobulin (Ig) E and the proliferation of eosinophils, thus exerting a critical role in regulating the development of skin diseases (Kasperska-Zajac et al., 2008; Kanda et al., 2019). Previous studies have shown that DHEA and cortisol probably regulate the cytokine network involved in chronic inflammatory and immune-mediated processes (Kasperska-Zajac et al., 2007; Buske-Kirschbaum et al., 2010). Therefore, cortisol and DHEA seem to be endogenous regulators involved in the development of skin diseases, such as PN, but such a phenomenon has not yet been determined. The behavior in the systemic circulation of PN patients has not been investigated. Therefore, in this study, we evaluated plasma concentrations of cortisol, cortisone, DHEA, testosterone, and progesterone in patients suffering from PN and in a matched control group.

## 2 Materials and Methods

### 2.1 Participants

This cross-sectional observational study was performed in the Department of Dermatology at a tertiary care hospital in Shenzhen, China, after approval from the institutional ethics committee. This study group consisted of 36 patients (19 males and 17 females; mean age 47.2 ± 9.3 years) diagnosed with PN by two independent dermatologists and 36 age- and gender-matched healthy controls (male/female 19/17; mean age 46.8 ± 9.1 years). All patients were diagnosed with PN by two independent dermatologist based on clinical features and histopathological findings. Clinically, PN is defined as the presence of numerous, pruritic and symmetrically distributed reddish-brown nodules. The skin lesions in all patients were on the extremities and trunk in this study. The administration of antihistamine drugs was discontinued approximately 2 weeks before the study. The participants taking any other medications affecting the levels of the hormones measured until 6 weeks into the study were excluded. Patients with skin infection or systemic disease were excluded. Use of systemic immunosuppressants or corticosteroids within the past 4 weeks, topical steroids or immunomodulators within the past 2 weeks, or limited use of moisturizers within the past 24 h prior to biopsy. All participants gave written, informed consent, and this study was approved by the Health Science Research Ethics Board of Southeast University and the Ethical Committee of Peking University Shenzhen Hospital (No. 20160427).

### 2.2 Measures

#### 2.2.1 Assessment of Prurigo Nodularis Symptoms

All PN patients were asked about their current pruritus severity (over the last 24 h) during the initial examination via questionnaires including four categories, the prurigo score (Siepmann et al., 2013) (PRUNOSI ranging 0–3), the visual analog scale (Aitken, 1969) (VAS, a graphic tool with a 100-mm horizontal line with the left end marked as “no symptom” and the right end marked as worst imaginable symptom), the verbal rating scale (Williamson and Hoggart, 2005) (VRS scores ranging 0–3, 0 = none, 1 = mild, 2 = moderate, 3 = severe), and the numerical rating scale (NRS scores ranging 0–10, 0 = no pruritus, 10 = worst imaginable pruritus). In addition, the dermatology life quality index (DLQI, total scores ranging from 0–30, 0–1 = no impairment in quality of life, 2–5 = mild impairment, 6–10 = moderate impairment, 11–20 = severe impairment, and 21–30 = very severe impairment) (Finlay and Khan, 1994) was also included.

### 2.3 Blood Sampling and Steroid Assay

Blood samples of all patients were collected between 8:00 and 10:00 a.m. and stored at −80°C until they were studied. After lightly applying a tourniquet, blood samples were drawn from the antecubital vein. They were immediately placed into clean tubes. To prevent clotting, heparin (14–17 IU/ml) was added to the tubes prior to sampling. Thereafter, the tubes with blood samples of approximately 2 ml were centrifuged at 3000 rpm for 5 min to separate blood cells and precipitate proteins. Then, 200 μl supernatant plasma was collected, processed and analyzed using high–performance liquid chromatography (Agilent 1200 HPLC system, Agilent, Waldbronn, Germany) and tandem mass spectrometry (ABI 3200 Qtrap, ABI, Foster City, CA, United States) (LC–MS/MS) (Chen et al., 2019; Chu et al., 2020). The method showed good linearity (*R* ^2^ > 0.99) in the range of 0.09–500 ng/ml, and the limits of quantitation (*LOQs*) were 0.1, 0.4, 0.3, 0.09, and 0.1 ng/ml for cortisol, cortisone, DHEA, testosterone, and progesterone, respectively. The coefficients of variation for the intraday and interday (*n* = 5) assays were less than 15%.

### 2.4 Statistical Analysis

The non-normal distribution of the data was examined by a one-sample Shapiro–Wilks test. Non-normally distributed data are expressed as the median and interquartile range (IQR). Comparisons between groups were conducted by a Mann–Whitney *U* test. Correlation was evaluated with the Spearman coefficient (*r*). A *p* value less than 0.05 was considered significant. All data analyses were performed using SPSS 26.0 (SPSS Inc., Chicago, IL, United States) for Windows.

## 3 Results

### 3.1 The Correlations Among the Scores of the Five Scales

The pruritus of PN is assessed by the four scales of PRUNOSI, VAS, NRS, and VRS. All the coefficients of Spearman’s correlations (*r*) between the four scales were no less than 0.75 (*p*s < 0.001), especially for the very high correlation between VAS and NRS (*r* = 0.93), as shown in Figure 1. These results showed that the four scales were highly consistent in the assessment of pruritus severity. In addition, the VAS, VRS, NRS, and PRUNOSI scores, which are indicative of pruritus severity, were all highly correlated with the DIQL scores (*r* = 0.87–0.97, *p*s < 0.001) (Figure 1).

**FIGURE 1:** A Spearman’s correlation coefficient (r) between the visual analog scale (VAS), numerical rating scale (NRS), verbal rating scale (VRS), the prurigo score (PRUNOSI), and dermatology life quality index (DLQI) among the PN patients (*n* = 36).

### 3.2 Comparison Between Prurigo Nodularis Patients and Controls in Levels of Plasma Steroids and Their Ratios

Median plasma concentrations of cortisol, cortisone and progesterone were significantly lower in PN patients as than in healthy subjects (*p*s < 0.05) (Figure 2). Median plasma concentrations of testosterone and DHEA were not significantly different in PN patients compared with healthy controls (*p* > 0.146). The PN patients showed significantly lower plasma levels of cortisone to cortisol (*p* < 0.01) and higher levels of testosterone to cortisol (*p* < 0.01) than healthy controls. There was no difference in DHEA to testosterone ratio between PN patents and controls (Figure 2).

**FIGURE 2:** Comparison of PN patients (*n* = 36) and controls (*n* = 36) in terms of steroids and their ratios in plasma.

The median plasma levels of testosterone and the ratios of testosterone to cortisol and DHEA in male PN patients were significantly higher than those in female PN patients (*p*s < 0.05). Plasma levels of progesterone and the DHEA to cortisol ratio in male PN patients compared with females were significantly lower (*p*s < 0.05) (Supplementary Table S1). The level of the ratio of cortisol to cortisone was marginally significantly higher in male PN patients than in female PN patients (*p* = 0.058), but this was not true for other steroids and ratios (*p*s > 0.196) (Supplementary Table S1).

### 3.3 Associations Between the Scales and Candidate Biomarkers Among Prurigo Nodularis Patients

Even further, among the candidate biomarkers (i.e., cortisol, cortisone, progesterone, the ratios of cortisone, and testosterone to cortisol) showing intergroup differences, the associations of the levels of these candidates with the scores of five PN-related scales were performed for the purpose of screening the biomarkers to evaluate the pruritus severity and quality of life of PN. The concentrations of plasma cortisol and cortisone showed highly (*p*s < 0.001, *r* = −0.84 to −0.94) or moderately (*p*s < 0.01, *r* = −0.43 to −0.62) negative correlations with all the scores of the four PN symptoms (i.e., PRUNOSI, VAS, NRS, VRS, and DLQI). There were moderately positively significant correlations of the ratios of cortisone and testosterone to cortisol with the scores of the five scales (*p*s < 0.05, *r* = −0.36 to −0.48). There was no significant correlation between progesterone and the five scales (*p*s > 0.126).

## 4 Discussion

In the present study, it was found that the levels of four out of the eight biomarkers, including cortisol, cortisone, the ratios of cortisone, and testosterone to cortisol, were abnormal in PN patients. These biomarkers were significantly different in plasma from patients with PN compared to healthy controls and were found to be related with PN symptoms, especially pruritus severity, thus showing that the four biomarkers could be used to assess the pruritus severity of PN. To the best of our knowledge, this was the first attempt to screen sensitive endocrine biomarkers for objectively assessing the pruritus severity of PN. This was also the first investigation to verify the influence of PN on the two neuroendocrine systems, including the HPA and HPG axes, as well as on the interactions between the two systems. However, in this study, the plasma concentrations of DHEA and testosterone did not differ significantly between PN patients and healthy controls.

The pathogenesis of AD and PN was suggested by previous observations of dermal hyperplasia of nerve fibers or increased skin levels of interleukin 31 (IL-31) in both PN and AD (Sugiura et al., 1997; Sonkoly et al., 2006). It has been shown that AD patients showed lower cortisol levels than healthy controls (Buske-Kirschbaum et al., 2010). Based on this study, the authors suggested that cortisol might be one of the regulators implicated in AD pathogenesis, controlling the secretion of interleukin (IL) 4 and IL-5, which are the stimulating factors in the early stage of AD by activating Th-2 (Liu et al., 2011). A pattern of decreased circulating blood cortisol concentrations was also observed in other skin diseases, such as chronic urticaria (Ucmak et al., 2014; Varghese et al., 2016). These findings showed that chronic skin diseases (e.g., PN and chronic urticarial) would lead to hypocortisolism of the central HPA axis. When exposed to acute stress temporary activation of the central HPA axis generally occurs, resulting in the secretion of cortisol and increased cortisol levels (Varghese et al., 2016). In contrast, chronic stress may lead to the continuous activation of the HPA axis, leading to a blunted central HPA axis, followed by a hypocortisolism and a cortisol decrease (Rui et al., 2014). Chronic skin diseases with itch-scratch behavior may accelerate and prolong the altered integrity of the skin barrier in PN as chronic stressors, leading to a lower secretion of cortisol, further resulting in a hypocortisolism of the central HPA axis. Indeed, a decreased plasma cortisol in PN patients compared with healthy controls was observed in our study (Figure 2). We also found that the plasma cortisone concentration was lower in PN patients than in healthy controls. This is because inactive cortisone in plasma mainly originates from active cortisol under the catalysis of 11*β*-hydroxysteroid dehydrogenase type 1 isozyme (11β-HSD1) (López Bernal et al., 1982). Previous studies have shown that cortisone levels were decreased in response to chronic stress (Blair et al., 2017; Lee et al., 2019). It has been shown that the peripheral HPA axis in the skin might be implicated in the etiopathogenesis of PN (Kim et al., 2013). Previous human studies have revealed that the peripheral HPA axis may have regulatory mechanisms equivalent to those of the central HPA axis, secreting corticotrophin-releasing hormone (CRH) and expressing CRH-R1 receptors in response to stress (Kim et al., 2013; Rui et al., 2014). However, these pathomechanisms involving the role of stress in the etiopathogenesis of PN need to be further validated in future research. In addition, the plasma concentrations of cortisol and cortisone were found to be significantly negatively related to the pruritus severity of PN (Figure 3). A recent study showed that cortisol and cortisone were negatively correlated with the severity of chronic urticarial disease (Lee et al., 2019). The anti-inflammatory effect of cortisol may be related to its antipruritic properties, which in turn promotes healing of itchy nodules. Currently, the mechanism of antipruritic action can only be speculated upon.

**FIGURE 3:** Spearman’s correlation coefficients between the five scale scores, the levels of steroids and their ratio in plasma in patients with PN (*n* = 36).

The effects of sex hormones, such as DHEA and testosterone, on the pathogenesis of skin diseases have been extensively studied in recent years. Reduced serum concentrations of DHEA and DHEA-S have been observed in chronic inflammatory diseases, suggesting a shift to cortisol at the expense of adrenal androgen (Sturgeon et al., 2014). Abnormal circulating sex hormone concentrations have been confirmed in both male and female AD patients. However, other studies concerning sex hormones in skin diseases have reported inconsistent results. For instance, a prior study demonstrated decreased serum DHEA in male patients with AD who suffered from mild to moderate skin lesions (Kasperska-Zajac et al., 2008). In our study, however, the plasma concentrations of DHEA and testosterone did not differ significantly between PN patients and healthy controls. Another study demonstrated no differences in serum concentrations of DHEA and testosterone between females with AD and controls (Kasperska-Zajac et al., 2007). In male PN patients, on the other hand, the plasma concentration of testosterone was significantly higher than those of the female PN patients, while plasma concentration of progesterone was significantly lower in male patients. There was no significant difference in the plasma concentration of DHEA between male and female PN patients (Supplementary Table S1). Data are scarce concerning the behavior of plasma concentrations of DHEA and testosterone in PN, and these results would deepen our understanding of the molecular mechanisms that are responsible for this disease. This notion needs to be confirmed in future research with a large-scale population.

A dysfunctional HPA axis will naturally lead to a dysfunctional HPG axis because both HPA and HPG axes secrete hormones that stimulate a reciprocal interaction between them (Chu et al., 2020; Chu et al., 2021). As a result, PN patients showed a decreased plasma concentration of progesterone compared with healthy controls (Figure 2), suggesting that hypocortisolism of the HPA axis is closely associated with impaired HPG axis activity among PN patients. This implied that PN patients might have abnormalities in the two endocrine systems, the HPA and HPG axes. The cortisone to cortisol ratio was used to evaluate the activity of 11β-HSD1 (López Bernal et al., 1982), and the interaction within the HPA axis (Jean et al., 2008; Wilson and Thayer, 2017). Accordingly, the reduced 11β-HSD1 activity was in PN patients along with the above-mentioned hypocortisolism of the HPA axis under chronic stress due to itching and pain of PN.

It has been demonstrated that elite athletes with long-term training stress showed lower cortisol to cortisone ratio, such as cyclists (Gatti et al., 2005). These results indicated that the ratio of cortisol to cortisone is a useful bioindicator of chronic stress. An increased testosterone to cortisol ratio was found in PN patients compared with healthy controls (Figure 2). It could likely hint that the interaction between the HPA and the HPG axis was enhanced in PN patients because they were used to evaluate the interaction of the HPA axis with the HPG axis. Researchers have demonstrated an increased testosterone-to-cortisol ratio in patients with higher psychopathy scores, demonstrating that there is an augmented interaction between the HPA and HPG axes (Glenn et al., 2011). Thus, it inferred that such a ratio would be related to PN-induced chronic stress, implicating the pruritus severity of PN patients. This assumption needs to be confirmed in future research with large-scale samples.

There were some limitations in this study. First, the small sizes may restrict the generalizability of our findings. Second, In this study, we used a cross-sectional design, so we cannot draw conclusions about causality and directionality. Finally, the lack of information concerning biopsy site location for PN samples is a limitation of this study. Despite these limitations, we present several findings about the PN physiological response in endocrine systems. Further research with larger-scale cohorts is needed to validate our findings.

## 5 Conclusion

In summary, this study is the first to report that greater pruritus severity is related to lower plasma concentrations of cortisol and cortisone among PN patients. In addition, we failed to detect significant differences between the concentrations of DHEA or testosterone in the peripheral blood of PN patients and the blood of matched controls.

## Data Availability

The original contributions presented in the study are included in the article/Supplementary Materials, further inquiries can be directed to the corresponding authors.
